The article "Mediating effect of mindfulness cognition on the development of empathy in a university context" was published in 2019. Journal: PLoS One.

# Mediating effect of mindfulness cognition on the development of empathy in a university context

**DOI:** 10.1371/journal.pone.0215569

**Published:** 2019-04-18

**Authors:** Raquel De la Fuente-Anuncibay, Ángela González-Barbadillo, Jerónimo González-Bernal, Esther Cubo, Juan P. PizarroRuiz

**Affiliations:** 1 Department of Science Education, University of Burgos, Castile and León, Spain; 2 Department of Health Sciences, University of Burgos, Castile and León, Spain; 3 Burgos University Hospital, Neurology Department, Castile and León, Spain; Stanford University, UNITED STATES

## Abstract

Numerous interventions propose mindfulness training as a means of improving empathy. Our aim is to analyse the relationship between mindfulness practice and empathy through the mediating process of trait mindfulness. This sample comprised 264 undergraduate students ($\bar{\text{x}}=24,13\;\text{years}$, SD = 11,39). The instruments used were Five Facet Mindfulness Questionnaire and Toronto Empathy Questionnaire. The indirect effect was calculated using 10.000 bootstrap samples for the bootstrap confidence intervals corrected for bias. Empathy improvement is mediated by changes in the cognitions derived from mindfulness (B = .346, p<.01). The direct effect of mindfulness practice on empathy disappears in presence of this mediator (B = .133, p>.05). Mindfulness interventions that aim to improve empathy should focus on three of its components; *observing*, *describing and nonreactivity to inner experience*. Given the significance of the results, the research must be extended to larger samples.

## Introduction

Over the past decade, mindfulness-based interventions have been seen to offer promising therapeutic results throughout the life cycle, from infancy to senescence [1–3].

Within this field, clinical and health-related studies enjoy the greatest proliferation, although at present mindfulness practice is becoming increasingly prevalent in other settings, such as organizations, schools and in the world of sport [4–8].

In contrast, research relating mindfulness and college studies is scarce. The current systematic reviews of scientific production over the last ten years (2007–2017), based on the Web of Science, indicate a total of 652 articles published in any language, of which 96 articles are related to Social Science Research within the field of education. However, the studies linking mindfulness to university students have dropped to a total of 23 articles in which a total of 3,835 students have participated [9].

In this field, some studies [10] demonstrate its effectiveness in promoting health and well-being in university students, increasing student life satisfaction and significantly reducing depression and anxiety. Improvements are also noted in knowledge retention [11], grades improvement, in the areas of reading and science, and test performance [12].

Regarding the concept of empathy, it can be defined as an important component of social cognition that contributes to our ability to understand and respond adaptively to the emotions of others, to succeed in emotional communication and to promote prosocial behavior [13].

While definitions have changed according to different approaches and perspectives, recent research emphasizes the distinction between cognitive and emotional components [14]. The agreement between researchers and theorists on the interrelated processes that contribute to empathy has been difficult, there is a lack of consensus on whether the processes related to empathy—perspective taking, sympathy, personal distress, emotional contagion, mind theory—are part of “affective insight into the feelings of another, or are facets of a central process required for empathic responding” [13].

The main theoretical contributions and research on empathy and its relationship with mindfulness show that the human being is born with a biological predisposition to be empathetic, being the environment in which one evolves the one that determines one’s level of development. Educating in empathy opens the possibility of moving towards a society of understanding [15].

At a biological level, Lutz et al. [16] found that practicing mindfulness affected the neuronal processes associated with empathic responses. Hölzel et al. [17] concluded that 30 minutes of daily meditation increased the grey-matter density of the parts of the brain associated with empathy. Along the same lines, the practice of mindfulness has also been related to a greater amount of grey matter in the part of the cerebellum associated with cardiorespiratory control [18].

Many studies indicate that training in mindfulness leads to an increase in the different aspects of empathic attitude [19]. Thus, mindfulness practice implies a change at the cognitive level in the different dimensions (observe, describe, act consciously …), and therefore in the cognitions of the *mindfulness* construct [20]. Research with therapists [21] concluded that those who practiced meditation scored higher for empathy than those that did not.

We found evidence of recent interventions that propose training in mindfulness as a means of working on and improving empathy [22–25] as it increases empathy responses [26].

However, some results suggest contradictions about its effects, and in this sense Dekeyser et al. [27] in their study of a sample of psychology students and their parents, observed a negative association between the level of mindfulness and personal discomfort, which led to questioning the beneficial effect on empathy. However, further research reinforces the positive results. Although studies are limited and many issues remain unresolved [23, 28] there is preliminary evidence of a positive association between mindfulness and empathy [29].

To date there have been many studies that attempt to explain this relationship through correlation and regression analyses [23–24]. However, we did not find any research that empirically considers the mediating effects of the cognitions derived from mindfulness in relation to empathy. Moreover, most of the studies relating mindfulness practice to empathy have been conducted in therapeutic contexts and focus on health variables or on how mindfulness improves therapists’ empathic skills [21, 30, 31]. It is not easy to find studies conducted in non-professionalized or non-therapeutic contexts that relate the two variables [32] and we haven’t found any paper that studies the mediating effects on the university population.

The main objective of this study is to further the understanding of why mindfulness practice impacts on empathic processes, by analyzing the mediating effects of the cognitions that derives from *mindfulness* construct. The study focuses on its practice in informal contexts or environments–during leisure activities, at meditation centers or in mindfulness-related courses–which have been largely ignored in previous studies.

We have conceptualized empathy as a mainly emotional process that does not depend on a cognitive understanding, although it is considered that it can facilitate both understanding and action [13].

Thus, in accordance with the results of other investigations, we hope to confirm that mindfulness practice improves empathy -hypothesis 1-. However, our hypothesis considered that this total effect would be mediated by the changes that practicing mindfulness engenders in the cognitions of the *mindfulness* construct. In other words, that mindfulness practice (conduct) modifies the mindfulness cognitions -hypothesis 2- and that this improves empathy (emotion) -hypothesis 3-, with the direct effect of mindfulness practice on empathy disappearing in the presence of this mediating variable -hypothesis 4-.

Afterwards, the indirect effects of each facet of mindfulness construct are studied to determine which mediators have the greatest impact in terms of improving empathy -hypotheses 5 to 7- through mindfulness practice.

## Methods

### Participants

A non-probabilistic convenience sample of 264 volunteer students from Sheffield Hallam University, South Yorkshire, England, was used. The gender distribution was 48 males and 216 females, from the Faculty of Psychology, with an average age of 24.13 years (SD = 11.39; age range = 18–71 years). With regard to the gender distribution, although there is a marked bias towards the female population, this proportion is representative of the university population in the field of studies analyzed, the OECD indicators [33] on higher education indicate that there are great differences according to the field of study, and the percentage of women in the United Kingdom in the area of education is 74%, Ireland (68%) and Spain (81%) with respect to the area of health and social services United Kingdom (79%), Ireland (75%) and Spain (72%). In this case we have chosen to have a larger representative sample of the population studied to the detriment of a more homogeneous sample.

With regard to the practice of mindfulness, the participants answered the following question: “Have you had any mindfulness training?”. Thus, the sample was divided into two groups: those who had never practiced mindfulness before and those who had practiced it in informal contexts, that is, outside closed programs with a predetermined number of sessions.

### Measures

The instruments used were the Five Facet Mindfulness Questionnaire, FFMQ [20] and Toronto Empathy Questionnaire, TEQ [13], selected for their psychometric characteristics and their appropriateness for the purpose of the study. In addition, both scales have been used in previous studies with a university population similar to that of this study [34–36]. The FFMQ was designed to measure mindfulness with psychometric guarantees through factor analysis encompassing five different scales that measure a trait-like general tendency to be mindful in daily life. The FFMQ comprises 39 items relating to five different subscales: observing (the ability to perceive and recognize internal or external stimuli), describing (labeling internal experiences with words), acting with awareness, non-judging of inner experience (referring to a dispassionate stance toward thoughts, sensations or emotions) and non-reactivity to inner experience (referring to how removed the subject is from their thoughts and feelings and how quickly or slowly they react to a stimulus). These are grouped into a general second-order factor that collects the cognitions of mindfulness in a single dimension. It provides a broader assessment of mindfulness in terms of attention control, emotion regulation and self-awareness compared to other popular scales such as the Mindful Attention Awareness Scale (MAAS) [37]. The FFMQ has been validated in several countries, languages and cultures such as France, Holland, Germany, China, Norway and Chile amongst others [38]. It is adequately reliable and has convergent and discriminant validity (Cronbach’s alpha of .75 to .92) [20].

Toronto Empathy Questionnaire. The TEQ [13] is a brief and reliable questionnaire (Cronbach’s alpha of .81) that measures empathy as a primary emotional process. From a compilation of the scales most commonly used to measure this construct, an exploratory factor analysis generated a unique one-dimensional factor of empathy. It has shown strong convergent validity, correlating positively with behavioral measures of social decoding and self-reported measures of empathy [13]. It comprises 16 unidimensional items representing a wide variety of empathy-related behaviors, including emotional contagion, the demonstration of appropriate sensitivity following assessment of emotional states in others, altruism, sympathetic physiological arousal and pro-social helping behaviors.

The detailed protocol can be found at: http://dx.doi.org/10.17504/protocols.io.w8qfhvw.

### Study design

Based on the internal validity of the study, quasi-experimental design is used, as an attempt to control the influence of extraneous variables on the results. According to the number of evaluations it is a transverse study, since the participants are evaluated in a single temporary moment.

### Procedure

The written informed consent of the study participants was obtained, ensuring the confidential treatment of the data collected. The purpose and characteristics of the research were explained to them. The students completed the questionnaires with an average time of 25–30 minutes. The team members collected the information in one phase. The study complied with the ethical values required in research with people, respecting the fundamental principles included in the Declaration of Helsinki, in its updates, and in the regulations in force. This study was specifically approved by the Bioethics Committee at the University of Burgos, Spain, (IR 15/2018).

## Results

The main objective of this work is to confirm, from the total measurement of the cognitions of the mindfulness construct, the relationship between practicing mindfulness (in informal contexts) and improving empathy.

To test the proposed model (Fig 1), we used the PROCESS macro for SPSS developed by Hayes [39] and specifically Model 4, a mediation model with one mediating variable. We based our analytical strategy on this procedure to evaluate the positive indirect effect of mindfulness practice on empathy through the mediating process of mindfulness cognitions. The indirect effect was calculated using 10,000 bootstrap samples for the bootstrap confidence intervals (CI) corrected for bias. An indirect effect is considered statistically significant if the CI established (95% CI) does not include the value 0. If the CI contains the value 0, the null hypothesis establishes that the indirect effect is equal to 0, i.e. that there is no association between the variables considered [34]. In addition, this technique allows the introduction of dichotomous variables into the model (in this case having practiced mindfulness or not), without the restrictions and disadvantages that others such as Structural Equation Modeling -SEM- (by means of Weighted Least Squares (WLS)-) present.

**Fig 1:** Hypothesized mediation model: Indirect effect of mindfulness practice on empathy through mindfulness cognition and total effect of independent variable on dependent variable.

The PROCESS macro (Model 4) was used to test Hypothesis 1, which established that mindfulness practice impacts on empathy.

For this hypothesis, the results reflecting the total effect of mindfulness practice (IV) on empathy (DV) confirm that practicing mindfulness improves empathy (B = .299, p<.001).

As regards Hypothesis 2, we also confirmed, as expected, that mindfulness practice improves mindfulness cognitions (B = .479, p<.001). Furthermore, as proposed in Hypothesis 3, the improvement in empathy relates to changes in mindfulness cognitions included in the FFMQ (B = .346, p<.001).

The results in respect of Hypothesis 4 suggest that the positive direct effect of mindfulness practice on empathy (B = .133, p = .088) disappears if the mediation of mindfulness cognitions in that relationship is taken into account, as considered in our exposition (Table 1).

**Table 1:** Mediation model (PROCESS, Model 4): Indirect effect of mindfulness practice of (IV) on empathy (DV) through changes in mindfulness cognition (mediating variable).

	B	SE	p
Mediating variable model (DV: Mindfulness cognition) Predictor			
Mindfulness practice	.479	.095	.0001
DV: Empathy Predictors			
Mindfulness cognition	.346	.055	.0001
Mindfulness practice (Direct effect)	.133	.088	.132
Total effect			
Mindfulness practice	.299	.090	.001
Indirect effect	B	BootSE	Boot 95% CI
Mindfulness practice → Mindfulness cognition → Empathy	.166	.047	[.087, .272]

IV = independent variable; DV = dependent variable; CI = confidence interval.

In Fig 2 we can observe the results of the mediation model, which indicate that the indirect effect is significant.

**Fig 2:** Results of the mediation model: Indirect effect of mindfulness practice on empathy through mindfulness cognition and total effect of independent variable on dependent variable (unstandardized regression coefficients) *** p<.001.

The second objective is to determine which facets of mindfulness play a mediating role in the total effect between practicing mindfulness and empathy.

To verify which dimensions of mindfulness play a mediating role in the relationship between mindfulness practice and empathy (Fig 3) we used the PROCESS macro for SPSS developed by Hayes [39] and specifically Model 4. As in the previous objective, the indirect effect was calculated using 10,000 bootstrap samples for the bootstrap confidence intervals (CI).

**Fig 3:** Hypothesized mediation model: Indirect effect of mindfulness practice on empathy through each mindfulness facets separately (H = hypothesis).

Table 2 presents the results of the indirect routes of mediation of each mindfulness facets separately.

**Table 2:** Mediation model (PROCESS, Model 4): Indirect effect of mindfulness practice (IV) on empathy (DV), presenting the mediating impact of each mindfulness facets separately (mediating variable).

Indirect effect	B	BootSE	Boot 95% CI
MP → Observing → Empathy	.136	.038	[.072, .224]
MP → Describing → Empathy	.101	.033	[.044, .178]
MP → Acting with awareness → Empathy	.024	.022	[-.006, .085]
MP → Non-judging of inner experience → Empathy	.100	.016	[-.008, .057]
MP → Non-reactivity to inner experience → Empathy	.096	.037	[.038, .186]

MP = Mindfulness Practice

As seen, only the indirect effects of the mediation models in which the mediating variables are observing, describing and non-reactivity to inner experience are significant. Therefore, we can consider that the facets acting with awareness and non-judging of inner experience do not play a mediating role in the relationship established between the practice of mindfulness and empathy.

Our analysis of the significant indirect effects (Fig 4) revealed that mindfulness practice impacts on observing (H1: B = .828, p<.001) and this in turn effects empathy (H2: B = .164, p<.001). Moreover, the positive direct effect of mindfulness practice on empathy (H3: B = .163, p = .075) disappears if the mediation of the observing facet in that relationship is taken into account.

**Fig 4:** Results of the mediation model: Indirect effect of mindfulness practice on empathy through each mindfulness facets separately (unstandardized regression coefficients) *** p<.001, * p<.05.

As regards Hypothesis 4, we found that mindfulness practice impacts on describing (B = .587, p<.001) and this capacity in turn impacts on empathy (H5: B = .164, p<.001). However, this mediation is partial, and the direct effect is significant (H6: B = .198, p = .025).

As regards Hypothesis 7, we found that mindfulness practice impacts on non-reactivity to inner experience (B = .557, p<.001), with a concomitant effect on empathy (H8: B = .173, p<.001). However, this mediation is also partial, and the direct effect is significant (H9: B = .203, p = .026).

## Discussion

The findings found in this paper seem to indicate that mindfulness practices in informal settings involve modifications in mindfulness cognition, and that these also influence the development of empathy.

Its importance and the confirmation of a positive relationship between both variables has been pointed out in the review carried out, although we intend to advance with the study of the mediating effects of mindfulness thought in relation to empathy. A growing body of research on the benefits of mindfulness has begun to show its potential as an intervention strategy for improving mental health and overall performance.

However, Shapiro et al [40] considers it necessary to identify the mechanisms of action that are the basis of mindfulness in order to determine whether its development is what really leads to the positive changes that have been observed in many fields.

In addition, research with university students points to the need to increase investigation into positive aspects of functioning [9].

The study presented aims to respond to both shortcomings, on the one hand to provide new data in the university and non-therapeutic field that reaffirm the importance of this relationship; and on the other hand, having detected the lack of studies on the mediating effects of mindfulness, to shed some light on the underlying process.

Numerous studies have found a correlation between the practice of mindfulness and empathy, yet most of the literature collects results from structured mindfulness programs, carried out in professional or therapeutic contexts applied mainly in health contexts [24], as well as in academic contexts like that of the present study [41–44].

The meta-analysis conducted by Konrath [45], which analyzes 72 studies on empathy on university students in the United States between 1979 and 2009, shows a 40% empathetic decrease in students from 30 years ago until today, which is detrimental to attitudes of understanding, compassion, concern or empathy towards other people.

Studies carried out applying a program of meditation among the university population [46] in order to test the effects of meditation on alexithymia and social skills, revealed significant differences in the social skills variable and in five of its post-test measures factors.

Barbosa et al. [32] have pointed to the effects of programs based on mindfulness to reduce anxiety and increase empathy in a sample of students; along the same lines Sierra et al. [8] have shown a decrease in school stress and an increase in empathy in high school students. Other works that relate both constructs [47] point to benefits and state that, even brief interventions—5-minute meditation -, improve empathic understanding and the ability to decode emotions and mental states from subtle facial signals.

The theoretical relationship between the two constructs could be in the Grossman et al. [48] definition of mindfulness: the ability to maintain attention from moment to moment on emotional and social events, which may be ours or others', and in a non-evaluative manner.

Concurring with Viciana et al. [9] on the current need to study aspects of positive functioning in the university sector, our results seem to confirm that these informal practices have an effect on trait mindfulness [20], and that this implies an improvement in their levels of empathy (Hypothesis 1 and 2). Moreover, in the presence of this mediator, the direct effect of the practice of mindfulness on empathy disappears (Hypothesis 4), confirming the total mediation of the cognitions of the mindfulness construct in this relationship (B = .166, BootSE = .047, Boot 95% CI = [.038, .186]).

The findings of the second objective indicate that the observing dimension is the most robust mediator between the practice of mindfulness and empathy. And, although to a lesser extent, the describing and the non-reactivity of the internal experience dimensions also mediate in this relationship.

Further work is therefore needed to establish that mindfulness programs that aim to improve empathy should focus on these three components.

One of the limitations of this work arises from the unequal gender distribution of the sample, in which there is a bias towards the female gender. However, as stated before, we consider that it is a sample that represents in its composition the distribution of the population studied.

Another possible limitation to the study derives from self-reported measures as the only measure for mindfulness and empathy, although the instruments used have proven reliability and validity and are constructed from a factorial analysis of the most relevant scales on both constructs. Some authors point out the difficulty of differentiating subjective perception or actual increase, and propose, for example, to complement the results by means of a situational assessment of empathy—using execution measures or biological markers such as oxytocin—in order to differentiate between exact and subjective empathy [19, 49] mindfulness behavioral measures [50] and/or objective monitoring of mindfulness practice [51].

## References

[1] CoholicDA, EysM. Benefits of an Arts-Based Mindfulness Group Intervention for Vulnerable Children. Child and Adolescent Social Work Journal, 2015 10.1007/s10560-015-0431-3

[2] TedKS, ChanHY, WeeST, GohLG, NurF, Ying TanCT, et al Mindful Awareness Practice (MAP) to improve the cognition of singaporean elderly with Mild Cognitive Impairment (MCI): a randomized controlled trial (rct). Alzheimer’s y Dementia. 2016 10.1016/j.jalz.2016.07.118

[3] ZengX, ChanV, LiuX, OeiTPS, LeungFYK. The Four Immeasurables Meditations: Differential Effects of Appreciative Joy and Compassion Meditations on Emotions. Mindfulness. 2017 10.1007/s12671-016-0671-0

[4] Bruno SolariM. Estudio exploratorio cualitativo sobre una intervención piloto de mindfulness en una organización en Santiago de Chile. Mindfulness y Compassion. 2016 10.1016/j.mincom.2016.09.004

[5] FrancoC, SorianoE, JustoE. Incidencia de un programa psicoeducativo mindfulness (conciencia plena) sobre el autoconcepto y rendimiento académico de estudiantes inmigrantes sudamericanos residentes en España. Revista Iberoamericana de Educación. 2010; 53: 6.

[6] Palmi i GuerreroJ, SoléS. Intervenciones basadas en Mindfulness (Atención Plena) en Psicología del Deporte. Revista de psicología del deporte, 2016; 25: 147–155.

[7] Schonert-ReichlK, LawlorM. The effects of a mindfulness-based education program on pre- and early adolescents’ well-being and social and emocional competence. Mindfulness. 2010 10.1007/s12671-010-0011-8

[8] SierraO, UrregoG, MontenegroG, CastilloC. Estrés escolar y empatía en estudiantes de bachillerato practicantes de Mindfulness. Cuadernos de Lingüística Hispánica. 2015; 26: 175–197.

[9] VicianaV, FernándezA, LinaresM, EspejoT, PuertasP, ChacónR. Los Estudios Universitarios y el Mindfulness. Una revisión Sistemática. Revista Iberoamericana sobre Calidad, Eficacia y Cambio en Educación. 2018 10.15366/reice2018.16.1.008

[10] DvorakovaK, KishidaM, LiJ, ElavskyS, BroderickPC, AgrustiMR, et al Promoting healthy transition to college through mindfulness training with first-year college students: Pilot randomized controlled trial. Journal of American College Health. 2017 10.1080/07448481.2017.1278605 28076182PMC5810370

[11] RamsburgJT, YoumansRJ. Meditation in the higher-education classroom: Meditation training improves student knowledge retention during lectures. Mindfulness.2014 10.1007/s12671-013-0199-5

[12] BakoshLS, SnowRM, TobiasJM, HoulihanJL, Barbosa-LeikerC. Maximizing mindful learning: Mindful awareness intervention improves elementary school students’ quarterly grades. Mindfulness. 2016 10.1007/s12671-015-0387-6

[13] SprengRN, McKinnonMC, MarRA, LevineB. The Toronto Empathy Questionnaire: Scale development and initial validation of a factor-analytic solution to multiple empathy measures. Journal of personality assessment. 2009 10.1080/00223890802484381 19085285PMC2775495

[14] RankinKP, KramerJH, MillerBL. Patterns of cognitive and emotional empathy in frontotemporal lobar degeneration. Cognitive Behavioral Neurology. 2005 10.1097/01.wnn.0000152225.05377.ab15761274

[15] Moya AlbiolL. La empatía. Entenderla para entender a los demás. 1^st^ ed Barcelona: Plataforma Actual; 2014.

[16] LutzA, Brefczynski-LewisJ, JohnstoneT, DavidsonRJ. Regulation of the Neural Circuitry of Emotion by Compassion Meditation: Effects of Meditative Expertise. PLoS ONE. 2008 10.1371/journal.pone.0001897 18365029PMC2267490

[17] HölzelBK, CarmodyJ, VangelM, CongletonC, YerramsettiSM, GardT, et al Mindfulness practice leads to increases in regional brain gray matter density. Psychiatry Research: Neuroimaging. 2010 10.1016/j.pscychresns.2010.08.006 21071182PMC3004979

[18] Vestergaard-PoulsenP, van BeekM, SkewesJ, BjarkamCR, StubberupM, BertelsenJ, et al Long-term meditation is associated with increased gray matter density in the brain stem. Neuroreport. 2009.10.1097/WNR.0b013e328320012a19104459

[19] Bellosta-BatallaM, Pérez-BlascoJ, CebollaA, Moya-AlbiolL. Empatía y Mindfulness. Convergencia teórica. Revista Latinoamericana de Psicología Positiva. 2017; 3: 34–44.

[20] BaerRA, SmithGT, HopkinsJ, KrietemeyerJ, ToneyL. Using Self-Report Assessment Methods to Explore Facets of Mindfulness. Assessment. 2006 10.1177/1073191105283504 16443717

[21] Wang SJ. Mindfulness meditation: Its personal and professional impact on psychotherapists. Dissertation, Capella University. 2007.

[22] FoukalMD, LawrenceEC, JenningsPA. Mindfulness and Mentoring Satisfaction of College Women Mentoring Youth: Implications for Training. Mindfulness. 2016 10.1007/s12671-016-0574-0

[23] FultonCL, CashwellCS. Mindfulness-based awareness and compassion: Predictors of counselor empathy and anxiety. Counselor Education y Supervision. 2015 10.1002/ceas.12009

[24] KrasnerMS, EpsteinRM, BeckmanH, SuchmanAL, ChapmanB, MooneyCJ, et al Association of an educational program in mindful communication with burnout, empathy, and attitudes among primary care physicians. JAMA. The Journal of the American Medical Association. 2009 10.1001/jama.2009.1384 19773563

[25] LamotheM, RondeauÉ, Malboeuf-HurtubiseC, DuvalM, SultanS. Outcomes of MBSR or MBSR-based interventions in health care providers: A systematic review with a focus on empathy and emotional competencies. Complementary Therapies in Medicine. 2016 10.1016/j.ctim.2015.11.001 26860797

[26] ShapiroSL, BrownKW, AstinJA. Toward the integration of meditation into higher education: A review of research. The Center for Contemplative Mind in Society 2008.

[27] DekeyserM, RaesF, LeijssenM, LeysenS, DewulfD. Mindfulness skills and interpersonal behaviour. Personality and Individual Differences. 2008 10.1016/j.paid.2007.11.018

[28] BibeauM, DionneF, LeblancJ. Can compassion meditation contribute to the development of psychotherapists’ empathy? A review. Mindfulness. 2016 10.1007/s12671-015-0439-y

[29] GreasonPB, CashwellCS. Mindfulness and Counseling Self-Efficacy: The Mediating Role of Attention and Empathy. Counselor Education and Supervision. 2009 10.1002/j.1556-6978.2009.tb00083.x

[30] Aiken GA. The potential effect of mindfulness meditation on the cultivation of empathy in psychotherapy: A qualitative inquiry. Dissertation, Saybrook University. 2006.

[31] MiróMT, IbáñezI, FelipeI, GarcíaNM. Entrenamiento en “Open Mindfulness”: Un Estudio Piloto. Revista de Psicoterapia. 2015; 26: 145–159.

[32] BarbosaP, RaymondG, ZlotnickC, WilkJ, ToomeyR, MitchellJ. Mindfulness-based stress reduction training is associated with greater empathy and reduced anxiety for graduate healthcare students. Education for Health. 2013 10.4103/1357-6283.112794 23823667

[33] OECD. Ministerio de Educación, Cultura y Deporte. Secretaría de Estado De Educación, Formación Profesional y Universidades Panorama de La Educación Indicadores de la OCDE 2016. Madrid: Secretaria General Técnica; 2016.

[34] SchmidtC, VinetEV. Atención Plena: Validación del Five Facet Mindfulness Questionnaire (FFMQ) en estudiantes universitarios chilenos. Terapia psicológica; 2015 7;33(2):93–102. Available from: 10.4067/s0718-48082015000200004

[35] QuezadaC, RobledoJP, RománD, CornejoC. Empatía y convergencia del tono fundamental. RLA Revista de lingüística teórica y aplicada; 50(2):145–65. Available from: 10.4067/s0718-48832012000200007

[36] MathadMD. Correlates and Predictors of Resilience among Baccalaureate Nursing Students. Journal of Clinical and Diagnostic Research [Internet]. JCDR Research and Publications; 2017; Available from: 10.7860/jcdr/2017/24442.9352PMC537683328384889

[37] ZhuangK, BiM, LiY, XiaY, GuoX, ChenQ, et al A distinction between two instruments measuring dispositional mindfulness and the correlations between those measurements and the neuroanatomical structure. Scientific Reports [Internet]. Springer Nature; 2017 7 24;7(1). Available from: 10.1038/s41598-017-06599-wPMC552468928740242

[38] RodríguezNS. Mindfulness: Instrumentos de evaluación. Una revisión bibliográfica. PSOCIAL; 2017; 3 (2): 46–65.

[39] HayesAF. Introduction to mediation, moderation and conditional process analysis: A regression-based approach. 1^st^ ed New York: Guilford Press; 2013.

[40] ShapiroSL, CarlsonLE, AstinJA, FreedmanB. Mechanisms of mindfulness. Journal of Clinical Psychology [Internet]. Wiley; 2006;62(3):373–86. Available from: 10.1002/jclp.2023716385481

[41] BirnieK, SpecaM, CarlsonLE. Exploring self-compassion and empathy in the context of mindfulness-based stress reduction (MBSR). Stress and Health [Internet]. Wiley; 2010 11 29;26(5):359–71. Available from: 10.1002/smi.1305

[42] ShapiroSL, BrownKW, ThoresenC, PlanteTG. The moderation of Mindfulness-based stress reduction effects by trait mindfulness: Results from a randomized controlled trial. Journal of Clinical Psychology [Internet]. Wiley; 2010 12 22;67(3):267–77. Available from: 10.1002/jclp.2076121254055

[43] BarbosaP, RaymondG, ZlotnickC, WilkJ, ToomeyRIII, MitchellJIII. Mindfulness-based stress reduction training is associated with greater empathy and reduced anxiety for graduate healthcare students. Education for Health [Internet]. Medknow; 2013;26(1):9 Available from: 10.4103/1357-6283.11279423823667

[44] GockelA, BurtonD, JamesS, BryerE. Introducing Mindfulness as a Self-Care and Clinical Training Strategy for Beginning Social Work Students. Mindfulness [Internet]. Springer Nature; 2012 8 3;4(4):343–53. Available from: 10.1007/s12671-012-0134-1

[45] Konrath S. Empathy: College students don’t have as much as they used to. University of Michigan News Service. 27 May 2010. https://news.umich.edu/empathy-college-students-don-t-have-as-much-as-they-used-to/

[46] De La FuenteM, FrancoC, SalvadorM. Efectos de un programa de meditación (mindfulness) en la medida de la alexitimia y las habilidades sociales. Psicothema. 2010; 22: 369–375.20667262

[47] TanLBG, LoBCY, MacraeCN. Brief mindfulness meditation improves mental state attribution and empathizing. PLoS ONE. 10.1371/journal.pone.0110510 25329321PMC4201548

[48] GrossmanP, NiemannL, SchmidtS, WalachH. Mindfulness-based stress reduction and health benefits. Journal of Psychosomatic Research [Internet]. Elsevier BV; 2004 7;57(1):35–43. Available from: 10.1016/s0022-3999(03)00573-715256293

[49] BreithauptF. Kulturen der empathie. 1^st^ ed Frankfurt am Main: Suhrkamp; 2009.

[50] GrossmanP. Defining mindfulness by how poorly I think I pay attention during everyday awareness and other intractable problems for psychology’s (re)invention of mindfulness: comment on Brown, et al. (2011). Psychological Assessment. 2011 10.1037/a0022713 22122674

[51] QuintanaM, RiveraO. Mindfulness training online for stress reduction, a global measure. Studies in Health. Technology and Informatics. 2012.22954845

